RETRACTED

# Ikzf2 Regulates the Development of ICOS^+^ Th Cells to Mediate Immune Response in the Spleen of *S. japonicum*-Infected C57BL/6 Mice

**DOI:** 10.3389/fimmu.2021.687919

**Published:** 2021-08-12

**Authors:** Shihao Xie, Haixia Wei, Anping Peng, Anqi Xie, Jiajie Li, Chao Fang, Feihu Shi, Quan Yang, He Huang, Hongyan Xie, Xingfei Pan, Xu Tian, Jun Huang

**Affiliations:** ^1^Department of Infectious Diseases, Key Laboratory for Major Obsteric Diseases of Guangdong Province, The Third Affiliated Hospital of Guangzhou Medical University, Guangzhou, China; ^2^State Key Laboratory of Respiratory Disease, Guangzhou Institute of Respiratory Health, The First Affiliated Hospital of Guangzhou Medical University, Guangzhou, China; ^3^Biological Resource Center, The Second Affiliated Hospital of Guangzhou University of Chinese Medicine, Guangzhou, China; ^4^College of Pharmacy, Guangzhou Medical University, Guangzhou, China; ^5^Key Laboratory of Immunology, Sino-French Hoffmann Institute, Guangzhou Medical University, Guangzhou, China

**Keywords:** *Schistosoma japonicum*, spleen, CD4^+^ T cells, ICOS, Ikzf2(Helios)

## Abstract

**Background:**

Th cells (helper T cells) have multiple functions in *Schistosoma japonicum* (*S. japonicum*) infection. Inducible co-stimulator (ICOS) is induced and expressed in activated T lymphocytes, which enhances the development of B cells and antibody production through the ICOS/ICOSL pathway. It remains unclear about the role and possible regulating mechanism of ICOS^+^ Th cells in the spleen of *S. japonicum*-infected C57BL/6 mice.

**Methods:**

C57BL/6 mice were infected with cercariae of *S. japonicum* through the abdomen. The expression of ICOS, activation markers, and the cytokine production on CD4^+^ ICOS^+^ Th cells were detected by flow cytometry (FCM) and quantitative real-time PCR (qRT-PCR). Moreover, the differentially expressed gene data of ICOS^+^ and ICOS^−^ Th cells from the spleen of infected mice were obtained by mRNA sequencing. Besides, Western blot and chromatin immunoprecipitation (ChIP) were used to explore the role of Ikzf2 on ICOS expression.

**Results:**

After *S. japonicum* infection, the expression of ICOS molecules gradually increased in splenic lymphocytes, especially in Th cells (*P* < 0.01). Compared with ICOS^−^ Th cells, more ICOS^+^ Th cells expressed CD69, CD25, CXCR5, and CD40L (*P* < 0.05), while less of them expressed CD62L (*P* < 0.05). Also, ICOS^+^ Th cells expressed more cytokines, such as IFN-γ, IL-4, IL-10, IL-2, and IL-21 (*P* < 0.05). RNA sequencing results showed that many transcription factors were increased significantly in ICOS^+^ Th cells, especially Ikzf2 (*P* < 0.05). And then, the expression of Ikzf2 was verified to be significantly increased and mainly located in the nuclear of ICOS^+^ Th cells. Finally, ChIP experiments and dual-luciferase reporter assay confirmed that Ikzf2 could directly bind to the ICOS promoter in Th cells.

RETRACTED

**Conclusion:**

In this study, ICOS^+^ Th cells were found to play an important role in *S. japonicum* infection to induce immune response in the spleen of C57BL/6 mice. Additionally, Ikzf2 was found to be one important transcription factor that could regulate the expression of ICOS in the spleen of *S. japonicum*-infected C57BL/6 mice.

## Introduction

Schistosomiasis is a disease caused by *Schistosoma* parasites in the human body. It is estimated that at least 229 million people required preventive treatment in 2018 (1). *Schistosoma japonicum* (*S. japonicum*) is the main epidemic *Schistosoma* in China. *S. japonicum* mainly infects the human body by the penetration of cercariae through the skin to cause disease (2). Once infected, the eggs released by *S. japonicum* is the major pathogenic substance, which can deposit on multiple organs (liver, etc.) in the body, causing damage, leading to liver fibrosis and splenomegalia (3). A variety of immune cells participate in the immune response caused by *S. japonicum* infection, and CD4^+^ T cells (Th cells) play an important role (4).

Although the pathological changes that occur in the liver after *S. japonicum* infection involved different molecular mechanisms have been extensively reported (5), splenomegaly and immune cell proliferation and activation induced by *S. japonicum* infection are now a focus of research on parasitic infections (6). However, the precise molecular mechanisms and transcriptional regulation corresponding to these cellular and immunological changes have not been fully confirmed.

*Schistosoma* worm eggs stimulate CD4^+^ T cells, which trigger a series of immune responses. After 5 to 6 weeks of *S. japonicum* infection, humoral immunity dominated by B cells plays a major role in anti-infection. It was reported that the inducible co-stimulator (ICOS)/ICOSL pathway promoted the formation of germinal centers, the maturation and development of B cells, and the production of specific antibodies (7, 8).

ICOS, a member of the CD28 family, which is expressed at low level on naive T cells, could be surged rapidly under the induction of CD3 plus CD28 activation signal (9). It is known that ICOS participates in the proliferation and differentiation of CD4^+^ T cells. In studies involving infection with *S. japonicum*, the expression of ICOS was significantly increased (3). Similarly, in *Trichinella spiralis* infection model, blocking ICOS resulted in a decrease in the expressions of TNF-α and the Th2 cytokines (e.g., IL-4 and IL-5) and the serum levels of total IgE. This result suggested that ICOS appears to be involved in the induction of both Th1 and Th2 immunity, but may be of heightened importance in Th2 responses (10). It was reported that when compared with wild-type control, *Mycobacterium tuberculosis* (Mtb)-infected ICOS^−/−^ mice showed lower bacterial burden during the late chronic stage of infection, and Th1 response against Mtb was increased, which was most likely to be caused by diminished numbers and frequencies of Tregs (11). The ICOS/ICOSL pathway enhances the expression of CD40L, which could bind to CD40 on B cells, and promotes B-cell differentiation, germinal center formation, and antibody class conversion (12).

RETRACTED

Based on the important regulatory role of ICOS in CD4^+^ T cells in the immune response, it becomes much valuable to find upstream genes that regulate the expression of ICOS. In the Th cells of systemic lupus erythematosus patients, the expression of ICOS in Th cells decreased by interfering with bcl-6 (13). The transcription factors of the Ikzf family are important to regulate the differentiation and development of early lymphocytes. Ikzf2 contains both an N-terminal zinc finger DNA-binding domain and a C-terminal zinc finger protein–protein interaction domain (14). The unique structure of Ikzf2 can directly bind the target DNA to play a regulatory role. The Ikzf family includes Ikaros (encoded by the gene *Ikzf1*), Helios (*Ikzf2*), Aiolos (*Ikzf3*), Eos (*Ikzf4*), and Pegasus (*Ikzf5*) (15). Knockout of the *Ikzf1* gene in mutant zebrafish causes defects in embryonic T-lymphocyte production and *Ikzf1* regulates embryonic T-lymphocyte production through Ccr9 and Irf4 (16). Knockout of the *Ikzf2* gene in fetal naive T cells impairs their ability to preferentially differentiate into Treg cells (17). In addition, *Ikzf3* can inhibit the expression of IL-2 and *Ikzf4* promotes the formation of Th1 cells and prevents the differentiation and development of Th17 (14). However, whether the Ikzf transcription factor family affects the function of CD4^+^ T cells by regulating the expression of ICOS is not clearly understood.

Herein, the characteristic of ICOS^+^ Th cells was investigated, and the mechanism of ICOS expressing on Th cells was explored in this study.

## Materials and Methods

### Mice

Female C57BL/6 wild-type mice (6–8 weeks old) were obtained from the Traditional Chinese Medicine University of Guangzhou Animal Centre (Guangzhou, China). All mice were maintained under specific pathogen-free conditions.

### *Schistosoma japonicum* Infections

Infected *Oncomelania hupensis* snails (purchased from the Chinese Institute of Parasitic Disease, Shanghai, China) were put into a cup of clean water, and then the shells were crashed with pliers. After keeping the snail in the water for about 1 h, a sterile loop was used to transfer the *S. japonicum* cercariae-containing water on a piece of clean cover slide, and the number of *S. japonicum* cercariae was counted under a microscope. The abdominal skin of mice was prepared by shaving, and then the cover slide with 40 ± 5 *S. japonicum* cercariae was put on the abdominal skin in close contact for 10 min. Mice were sacrificed at 5–6 weeks after infection. Animal experiments were performed in strict accordance with the regulations for the Administration of Affairs Concerning Experimental Animals, and all efforts were made to minimize suffering.

RETRACTED

### Reagents and Antibodies

RPMI 1640, Dulbecco’s modified Eagle’s medium (DMEM), FBS, penicillin, and streptomycin were obtained from Invitrogen (Grand Island, NY, United States). Red blood cell (RBC) lysis buffer (Cat: C3702-500ml) was obtained from Beyotime Biotechnology (Shanghai, China). The LB broth (Cat: SD7002) was obtained from Sangon Biotech (Shanghai, China). Ampicillin (Cat: MCR003) was obtained from Dingguo Biotech (Beijing, China). The following fluorescein-conjugated anti-mouse antibodies were obtained from BD and Biolegend: FITC-CD3 (145-2C11), APC-cy7-CD8 (54-6.7), Percp-cy5.5-CD4 (GK1.5), Percp-cy5.5-CD19 (6D6), APC-CD62L (MEL-14), APC-PD-1 (29F.1A12), PE-cy7-ICOS (C398.4A), Brilliant Violet 421-CD69 (H12F3), PE-CD25 (BC96), BV421-CXCR5 (J252D4), PE-CD40L (MR1), APC-IFN-γ (XMG1.2), PE-IL4 (11B11), PE-IL10 (JES5-16E3), PE-IL2 (JES6-5H4), APC-IL21 (FFA21), APC-IL5 (TRFK5), eFlour660-IL13 (Blo13A), APC-CD45 (30-F11), and anti-mouse CD16/CD32 (2.4G2). The eFluor506-FVD (Cat: 65-0863-14) was obtained from eBioscience. The Alexa Fluor 488 anti-rabbit IgG (Cat: 4412S), Helios rabbit mAb (D8W4X), histone H3 rabbit mAb (D1H2), α-tubulin antibody (Cat: 2144S), and HRP-conjugated secondary antibodies (Cat: L3012-2) were obtained from Cell Signaling Technology.

### Cells

Human embryonic kidney (HEK) 293T cells were grown in DMEM containing 10% heat-inactivated fetal bovine serum at the temperature of 37°C and in a 5% CO_2_ incubator (ESCO-CCL-170B-8, Suzhou, China).

### Splenic Lymphocyte Isolation

Mice were sacrificed and peripheral blood was collected after 5–6 weeks of infection. Then, the spleen from the mouse was obtained in a biological safety cabinet, and it was ground by a sterile syringe piston and filtered with a 100-μm filter. Then, the cell suspension was processed by using RBC lysis buffer and isolated cells were washed twice with HBSS (Hank’s balanced salt solution). Finally, lymphocytes were resuspended with 10% FBS RPMI 1640 for the following experiments.

RETRACTED

### Hepatic Lymphocyte Isolation

The liver of mouse was perfused with PBS solution to clear the peripheral blood and the liver was separated in a biological safety cabinet. The hepatic tissue was cut into small pieces (removal of the gallbladder) and processed with digestion buffer (collagenase IV) for 60 min at 37°C. Digested hepatic tissue was ground by a sterile syringe piston and filtered with a 100-μm filter. Cell suspension was processed by using RBC lysis buffer for 10 min. Next, 70% Percoll and 40% Percoll were prepared to separate lymphocytes. Isolated lymphocytes were washed twice with HBSS. Finally, lymphocytes were resuspended with 10% FBS RPMI 1640 for the following experiments.

### Pulmonary Lymphocyte Isolation

The lung of mouse was perfused with PBS solution to clear the peripheral blood and the lung was separated in a biological safety cabinet. Then, the lung tissue was cut into small pieces and was digested by digestion buffer (including collagenase IV and DNase I) for 30 min at 37°C. Digested lung tissue was ground by a sterile syringe piston and filtered with a 100-μm filter. Then, the cell suspension was processed by using RBC lysis buffer for 10 min and the isolated cells were washed twice with HBSS. Finally, lymphocytes were resuspended with 10% FBS RPMI 1640 for the following experiments.

### Detection of Peripheral Blood Leukocytes and Serum Transaminase

The peripheral blood in normal mice and infected mice was collected by EDTA-containing tubes. Peripheral blood serum in normal mice and infected mice was collected by coagulant-containing tubes. These samples were detected in the Laboratory Department of the Sixth People’s Hospital of Panyu District (Guangdong Province, China).

### Cell Surface Staining

The target cells were washed twice with PBS and blocked in PBS buffer containing 1% BSA for 30 min. Then, cells were stained with conjugated antibodies that were specific for cell surface antigens for 30 min at 4°C in the dark. The stained lymphocytes were detected by FCM (Beckman Coulter, Fullerton, CA, United States), and the results were analyzed with the software CytoExpert 2.3 (Beckman Coulter).

### Intracellular Cytokines and Transcriptional Factors Staining

The spleen cell suspension of each treatment group was stimulated with PMA (20 ng/ml, Sigma) and ionomycin (1 µg/ml, Sigma) in a 37°C, 5% CO_2_ incubator for 5 h with brefeldin A (10 µg/ml, Sigma) added in the last 4 h of incubation. Then, target cells were first stained with cell surface staining antibodies as described above. After that, cells were fixed with fixation and permeabilization solution (BD Biosciences) for 20 min at 4°C in the dark and permeabilized overnight at 4°C in PBS buffer containing 0.1% saponin (Sigma), 1% BSA, and 0.05% NaN_3_. When the samples were stained for transcription factors, no cell stimulation step is required. Next, cells were stained with conjugated antibodies that were specific for transcriptional factors and cytokines. The stained lymphocytes were detected by FCM (Beckman Coulter), and the results were analyzed with the software CytoExpert 2.3 (Beckman Coulter).

RETRACTED

### Flow Cytometric Sorting

Lymphocytes were resuspended by 10% FBS RPMI 1640 and stained with fluorescein-conjugated antibodies that were specific for cell surface antigens (such as C45, CD3, CD4, and ICOS) for 30 min at 4°C in the dark. Then, a fluorescence-activated cell sorting machine (FACS Aria cell sorter) (BD, Mountain View, CA, United States) was used to sort CD4^+^ ICOS^+^ and CD4^+^ ICOS^−^ cells.

### Magnetic Bead Sorting

Lymphocytes were resuspended twice in the sorting buffer and centrifuged to remove the supernatant. An appropriate amount of sorting buffer and specific magnetic bead-conjugated antibodies were added to the cells and incubated at 4°C for 30 min. Before sorting, the separation column was first rinsed with the sorting buffer. Then, the antibody-conjugated cells were injected into the columns and washed twice by the sorting buffer. Finally, the magnetic field was eliminated, the target cells were collected, and the purity of the target cells was detected by FCM.

### RNA Sequencing

Flow cytometric sorting was used to isolate ICOS^+^ and ICOS^−^ cells from the spleen suspension cells after *S. japonicum* infection. Then, the target cells were preserved by TRIzol and sent to Lianchuan Biological Company (Hangzhou, China) for RNA sequencing. Differentially expressed genes were the summary of upregulated and downregulated genes between samples. In this study, fold change (FC) ≥2 or FC ≤0.5 (the absolute value of log2FC ≥1) and the *P*-value <0.05 were used as the standard to evaluate the differentiation.

### Quantitative Real-Time PCR

Cell samples were cryopreserved with TRIzol (including suspended lymphocytes and sorted cells). Then, RNA was extracted by using chloroform, isopropanol, and 75% ethanol. cDNA was synthesized from total RNA by using SuperScript III Reverse Transcriptase (Takara, Cat: RR037A). Quantitative real-time PCR (qRT-PCR) was performed with a CFX96 Real-Time PCR Detection System by using TB Green Premix Ex Taq™ (Tli RNaseH Plus) (Takara, Cat: RR420A). Data were normalized by the *β-actin* and target gene-specific primers (**Table 1**).

RETRACTED

**Table 1:** Sequences of primers.

Gene	Forward primer	Reversed primer
*Bcl-6*	GACGCACAGTGACAAACCAT	AACTGCGCTCCACAAATGTT
*Maf-b*	GCGCACCTGGAAGACTACTA	GCATAGCCATCGGAAGCCAC
*C-maf*	CTGCCGCTTCAAGAGGGTGCAGC	TCGCGTGTCACACTCACATG
*Ikzf2*	TGAGAGACCTGCTGTCATAGA	CTGGGTAGCTGAATCGCATAA
*ICOS*	ACCAAGGGAAGCGGAAATG	GGAGCTGTCTGGGTTGTTTAG
*ICOS promoter*	GGACTCTAACCTCCCTTCAAATC	ATGTCAGCACACCCTGTTAC
*Gata-3*	GGCCAGGCAAGATGAGAAAG	AGGGCGGATAGGTGGTAATG
*β-actin*	CCGTAAAGACCTCTATGCCAAC	GGGTGTAAAACGCAGCTCAGTA

### Western Blot

CD4^+^ ICOS^+^ and CD4^+^ ICOS^−^ samples were obtained by flow cytometric sorting from *S. japonicum-*infected splenic lymphocytes. Nuclear and Cytoplasmic Protein Extraction Kit (P0027, Beyotime, China) was used to extract nuclear proteins and cytoplasmic proteins from the above cells. The protein samples were separated in 10% SDS-denatured polyacrylamide gel and transferred onto polyvinylidene difluoride membranes. Then, the membranes were blocked with 10% BSA-PBST at room temperature for 1–2 h. The membranes were incubated with Ikzf2 (Cst, Cat: 42427S), H3 (Cst, Cat: 4499S), or tubulin (Cst, Cat: 2144S) at 4°C overnight and then incubated with HRP-conjugated secondary antibodies (Cst, Cat: L3012-2) and detected with Clarity Max ECL Substrate (Cat: 170-5061).

### Chromatin Immunoprecipitation

The target cells are cross-linked with 1% formaldehyde and subsequently quenched with glycine. Then, cells were washed twice in cold 1× PBS and collected by centrifugation at 200*g*, 4°C. Nuclei preparation and chromatin shearing were completed by using truChIP^®^ Chromatin Shearing Kit (Covaris, Cat: PN 520127). DNA agarose electrophoresis was used to determine whether the chromatin shearing length was within the appropriate range. After chromatin shearing, 2% input sample was taken out. Then, SimpleChIP^®^ Plus Enzymatic Chromatin IP Kit (Magnetic Beads: 9005) was used to perform chromatin immunoprecipitation (ChIP), and the final results were evaluated by qRT-PCR.

### Plasmid Construction

PmirGLO plasmid containing the *ICOS promoter*, *luciferase*, and *hRluc* genes; pCDNA3.1(+) plasmid expressing the *Ikzf2* gene; and the corresponding empty vector were from Tsing Ke Bio-Tech (Beijing, China). All expression plasmids were ampicillin resistant and validated by Tsing Ke Bio-Tech.

### Plasmid Amplification and Extraction

Liquid LB media containing ampicillin (100 μg/ml) were used to amplify the competence containing the target plasmids. The culture media were placed in a shaker at 37°C, 250 r/min for 16–18 h. Then, the plasmids were extracted *via* Endo-free Plasmid Mini Kit I (Omega Bio-Tek, Guangzhou, China, Cat: D6948-01).

RETRACTED

### Plasmid Transfection and Dual-Luciferase Reporter Assays

HEK293T cells were placed on a 24-well plate (3 × 10^5^ cells per well) and cultured for 24 h. When the cell density was 70%–80%, the cells were transfected with plasmids using Lipofectamine 2000 (Invitrogen, cat: 11668-027) for 24 h. Then, the cells were lysed for dual-luciferase reporter assays (DLR) and Western blot detection. Briefly, the media were removed and the cells were added to the lysis buffer. Cell lysates were divided into two parts: one part was used for the DLR test, and the other part was used for protein expression of the transfected plasmid by Western blot. The luciferase activity was assessed using a Luciferase Reporter Assays Kit (Yeasen Bio-Tek, Shanghai, China, Cat: 11402ES60) by a GloMax Discover machine (Promega, Madison, United States).

### Statistical Analysis

Differences between the two groups were analyzed in GraphPad Prism (v8.02) using unpaired *t*-tests with equal variance and normal distributions. To compare more than two groups, one-way ANOVA and LSD test by SPSS software package and GraphPad Prism (v8.02) were used with equal variance and normal distributions. The Mann–Whitney *U* test was used when the data have unequal variance or non-normal distribution. Statistical significance was defined as *P <*0.05.

## Results

### *S. japonicum* Infection Induces Increased Expression of ICOS Molecules in Th Cells in the Spleen

In the mice model of *S. japonicum* infection, when compared with the naive group, the absolute number of lymphocytes in the spleen increased significantly after infection (*P* < 0.001, **Figure 1A**). Splenic lymphocyte suspensions expressed higher levels of ICOS mRNA than those from naive mice (*P* < 0.05, **Figure 1B**) and more splenic lymphocytes expressing ICOS in the infected mice (*P* < 0.01, **Figure 1C**). As shown in **Figure 1D**, when compared with the naive group, the proportion of ICOS^+^ Th cells was significantly increased in *S. japonicum*-infected mice (*P* < 0.01). Interestingly, the percentage of ICOS expressing B cells (CD3^−^ CD19^+^) in the infected mice was also higher than in naive mice (*P* < 0.05). No significant differences of ICOS expression in CD3^+^ CD8^+^ T cells were observed between naive and infected mice (*P* > 0.05).

**Figure 1:** *Schistosoma japonicum* infection-induced increased expression of ICOS molecules in Th cells in the spleen. Female C57BL/6 mice were infected with 40 ± 5 *S. japonicum* cercariae per mouse, and 5–6 weeks after infection, mice were euthanized. **(A)** Number changes of splenic lymphocytes in the naive group and *S. japonicum* infection group. Each group included six mice. **(B)** Transcriptional expression of ICOS from splenic lymphocytes of naive and *S. japonicum*-infected mice was detected by qRT-PCR. Each group included six mice. **(C)** The ICOS expression on mononuclear cells from naive and *S. japonicum*-infected mice was detected by flow cytometry. All the doublet cells, dead cells, and nonlymphoid cells were excluded from flow cytometry data. The control group is the fluorescence minus one (FMO) control. **(D)** ICOS expression on CD4^+^ Th cells, CD8^+^ T cells, and CD19^+^ B cells from naive and infected mice was detected by FACS. **(E)** ICOS^+^ cells from WT and infected mice mononuclear cells were gated firstly. The distributions of ICOS in different cell populations were shown. Data are representative of three experiments. **(F)** Dynamic changes of ICOS expression in CD4^+^ T cells from week 1 after infection; naive control was set (0 week). The average of three independent experiments with five to six mice per group was shown and repeated three times with similar results. The error bars are SD, *P < 0.05, **P < 0.01, ***P < 0.001, and *ns*, not significant (*P* > 0.05).

RETRACTED

At the same time, the changes in the proportions of various immune cells in splenic ICOS^+^ cells after *S. japonicum* infection were explored. Results (**Figure 1E**) showed that the proportion of ICOS^+^ Th cells was increased after *S. japonicum* infection. The proportions of CD3^+^ CD8^+^ ICOS^+^ T cells and other immune cells were not significantly changed in *S. japonicum*-infected mice *versus* naive mice. In contrast, the proportion of B cells in ICOS^+^ cells was reduced remarkably after *S. japonicum* infection.

Then, we investigated the dynamic change of splenic ICOS^+^ Th cells from week 1 to week 6 of *S. japonicum-*infected mice. As shown in **Figure 1F**, the percentage of splenic ICOS^+^ Th cells was remarkably increased from week 1 after *S. japonicum* infection and continued to increase in the course of infection and maintained at a high level from week 4 to week 6. These results suggested that *S. japonicum* infection could induce the expression of ICOS molecules in Th cells in the spleen. In addition, ICOS^+^ Th cells continue to increase and stay at the peak at 4–6 weeks after infection.

### The State and Cytokine Expression Profiles of Splenic ICOS^+^ Th Cells in *S. japonicum*-Infected Mice

The state of infected splenic ICOS^+^ Th cells was determined by measuring the CD25, CD69, and CD62L molecule expression with different fluorescence-labeled antibodies. As shown in **Figure 2A**, FVD^−^ CD45^+^ lymphocytes were gated firstly. Then, Th cells were gated, and the expressions of CD25, CD69, and CD62L on ICOS^+^ cells were detected. The result (**Figure 2B**) showed that the percentage of CD62L expressing ICOS^+^ Th cells in the infected group decreased significantly when compared with the naive group (*P* < 0.01). It was found that less ICOS^+^ Th cells expressed CD62L (*P* < 0.01) than CD4^+^ ICOS^−^ T cells in both the naive and infected groups. More ICOS^+^ Th subsets expressed CD69 (*P* < 0.01), and CD69^+^ ICOS^+^ Th cells significantly increased after *S. japonicum* infection (*P* < 0.01). There was no significant difference in the expression of CD25 between ICOS^+^ Th and ICOS^−^ Th cells from the naive and infected groups (*P* > 0.05). However, when compared with naive mice, more ICOS^+^ Th cells expressed CD25 in the infected group (*P* < 0.01). Next, the expressions of CXCR5 and CD40L, which are related to ICOS pathway function, were examined after *S. japonicum* infection. As shown in **Figure 2C**, the percentage of CXCR5^+^ cells in ICOS^+^ Th cells was significantly higher than that in ICOS^−^ Th cells from both the naive and infected mice (*P* < 0.01), and CXCR5 significantly increased in ICOS^+^ Th subsets after *S. japonicum* infection (*P* < 0.01). Interestingly, more ICOS^+^ Th subset in infected mice, not ICOS^+^ Th subset in naive mice, expressed CD40L than the corresponding ICOS^−^ Th group (*P* < 0.01). These results implied that CD4^+^ T cells expressing ICOS possess a stronger ability to activate and promote subsequent immune response after *S. japonicum* infection.

RETRACTED

**Figure 2:** The higher percentage of activation-associated molecules and cytokines expressed on splenic ICOS^+^ Th cells. Five to 6 weeks after *S. japonicum* infection, splenocytes were isolated, stained by different fluorescence-labeled antibodies, and detected by FACS. **(A)** All flow cytometry results were analyzed based on removing adhesions, elimination of dead cells, and gating on CD45^+^ CD3^+^ CD4^+^ populations. **(B)** Differences in activation markers of ICOS^−^ Th cells and ICOS^+^ Th cells in infected mice and naive mice. **(C)** The expression differences of functionally related surface markers in the two groups. **(D)** Splenocytes were stimulated by PMA and ionomycin, and intracellular cytokine staining was done. The CD4^+^ Th cells were gated firstly, and the expression of IFN-γ, IL-2, IL-4, IL-5, IL-10, IL-13, and IL-21 on ICOS^+^ cells was shown. Moreover, the cytokines expressed in the ICOS^−^ and ICOS^+^ cells were compared between naive and infected mice. The average of three independent experiments with five to six mice per group was shown and repeated three times with similar results. The error bars are SD, *P < 0.05, **P < 0.01 and *ns*, not significant (*P* > 0.05) compared with naive controls.

RETRACTED

Next, splenocytes were stimulated by PMA plus ionomycin, and intracellular cytokine staining was done to examine the cytokine-producing ability of splenic ICOS^+^ Th cells. As shown in **Figure 2D**, more ICOS^+^ Th subsets expressed IL-4, IFN-γ, IL-10, and IL-2 than the corresponding ICOS^−^ Th groups (*P* < 0.01). The proportion of IL-4-expressing ICOS^+^ Th cells in the infected group was higher than that in the naive group (*P* < 0.01). Similarly, the percentage of IL-10, IL-13, and IL-21 expressing CD4^+^ ICOS^+^ T cells in the infected group was also higher than that in the naive group (*P* < 0.05). It was also found that more ICOS^+^ Th subset in infected mice, not ICOS^+^ Th subset in naive mice, expressed IL-21 than the corresponding negative group (*P* < 0.05). Then, the percentages of IL-13 and IL-21 expressing ICOS^+^ Th cells in the infected group were higher than those in the naive group (*P* < 0.05). However, there was no significant difference in IL-5 expression between ICOS^+^ **^/^** ^−^ cells from the infected and naive groups (*P* > 0.05). These results indicated that ICOS^+^ Th cells from *S. japonicum*-infected mice produce more cytokines to regulate the immune response against *S. japonicum* infection.

### Differences in Genes Expression Between ICOS^+^ Cells and ICOS^−^ Th Cells After *S. japonicum* Infection

To investigate the upstream regulation mechanism of ICOS^+^ Th cells with *S. japonicum* infection, RNA sequencing was performed for flow cytometric sorted CD4^+^ ICOS^+^ T and ICOS^−^ Th cells from infected mice. The purity of target cells for RNA sequencing is shown in **Figure 3A**. When compared with ICOS^−^ Th cells, there were 508 upregulated genes and 781 downregulated genes in ICOS^+^ Th cells after *S. japonicum* infection (**Figure 3B**). To fully understand the selected genes, Gene Ontology (GO) and Kyoto Encyclopedia of Genes and Genomes (KEGG) analyses (**Figures 3C, D**) were conducted and the results showed that multiple selected genes were significantly enriched (*P* < 0.05). Data showed that ICOS participated in a variety of biological processes and had an important and complex function, such as DNA binding, immune system process, and immune response (**Figure 3C**). KEGG analysis (**Figure 3D**) showed that ICOS participates in a variety of signaling pathways, such as hematopoietic cell lineage, cytokine–cytokine receptor interaction, T-cell receptor signaling pathway, and Th1 and Th2 cell differentiation (*P* < 0.05). It indicated that ICOS was of great significance for the early differentiation of hematopoietic cells, lymphocyte maturation, and cytokine production. As shown in **Figure 3E**, the expressions of some activated markers in ICOS^+^ Th cells, such as CD69, CXCR5, PD-1, and CD40L, were higher than ICOS^−^ Th cells, which were consistent with the above FCM results (**Figure 2**). Furthermore, the expression of some chemokine receptors (CCR3, CCR4, CCR5) and immunomodulatory molecules (Tight, CTLA4, lLAG-3) was also higher in ICOS^+^ Th cells than that in the ICOS^−^ Th cells. Then, we explored the expression of cytokines from the two groups of cells. Unexpectedly, ICOS^+^ Th cells not only expressed more IL-4, IL-21, IL-10, and IFN-γ, but also expressed more TNF super family factors, such as TNFSF4, TNFSF11, TNFSF14, and TNFSF9 (**Figure 3F**). These results implied that ICOS expressing Th cells played multiple and complex roles in *S. japonicum*-infected mice.

RETRACTED

**Figure 3:** Different RNA expression between ICOS^+^ and ICOS^−^ splenic Th cells. Five to 6 weeks after *S. japonicum* infection, splenocytes were isolated and stained by different fluorescence-labeled antibodies. **(A)** CD3^+^ CD4^+^ ICOS^+^ T cells and CD3^+^ CD4^+^ ICOS^−^ T cells were sorted by FACS, and the purification was identified by FACS. RNA was extracted from these two purified cell populations, respectively. RNA sequencing was done. **(B)** Differentially expressed genes in CD4^+^ ICOS^−/+^ Th cells were shown. **(C)** GO enrichment analysis of differentially expressed genes in ICOS^−/+^ Th cells was shown. **(D)** KEGG enrichment scatter plots of differentially expressed genes in ICOS^−/+^ Th cells were shown. **(E)** Differences of surface molecule expression in ICOS^−/+^ Th cells were shown. **(F)** Differences of cytokine expression in ICOS^−/+^ Th cells were shown.

### Ikzf2 Was Highly Expressed in ICOS^+^ Th Cells From *S. japonicum*-Infected Mice

To further explore the upstream genes that regulate the expression of ICOS molecules, the differentially expressed transcription factors from the sequencing data were compared. As shown in **Figure 4A**, the expression levels of Ikzf2 and Ikzf4 were significantly increased in ICOS^+^ Th cells. Interestingly, the expression levels of bcl-6, maf, and tox2, which regulate the expression of Tfh cells, were also significantly increased in ICOS^+^ Th cells. Next, the differential expression of transcription factors was verified by qRT-PCR. These results were consistent with the results from mRNA sequencing (**Figure 4B**). The FC values of each member of the Ikzf transcription factor family are shown in **Figure 4C**, and it was found that the FC value of transcription factor Ikzf2 was the highest. Finally, the expression of Ikzf2 was detected in Th cells by FCM (**Figure 4D**). Data showed that the expression of Ikzf2 in ICOS^+^ Th cells was significantly higher than that in ICOS^−^ Th cells (*P* < 0.01). These results implied that Ikzf2, as a transcription factor regulating the early differentiation and development of T cells, may regulate the expression of ICOS in Th cells.

RETRACTED

**Figure 4:** Transcription factor Ikzf2 is highly expressed in ICOS^+^ Th cells. **(A)** The expressions of ICOS activation- and function-related transcription factors in ICOS^−/+^ Th cells detected by mRNA sequencing were compared. **(B)** ICOS activation function-related transcription factor differences were detected by qRT-PCR. **(C)** The comparison of the expression of Ikzf2 family members in CD4^+^ ICOS^+^ and CD4^+^ ICOS^−^ groups. FC (fold change) was the result after FPKM.ICOS^+^ **/**FPKM.ICOS^−^. Differential genes were selected based on FC ≥2, or ≤0.5, and *P* < 0.05. **(D)** The expression difference of Ikzf2 in CD4^+^ ICOS^−/+^ Th cells was detected by flow cytometry. All the doublet cells, dead cells, and nonlymphoid cells were excluded from flow cytometry data. Data are shown as three samples in each group from one representative experiment, and experiments were repeated three times with similar results. *P < 0.05, **P < 0.01.

### Ikzf2 Entered Into the Nucleus of ICOS^+^ Th Cells and Bound to the Promoter of ICOS Gene After *S. japonicum* Infection

To determine the role of Ikzf2 in inducing the expression of ICOS in Th cells, both the ICOS^+^ and ICOS^−^ Th cells were sorted by FACS. The cytoplasmic and nuclear proteins of the sorted cells were isolated and tested by Western blot to study the distribution of Ikzf2 after *S. japonicum* infection. Western blot analysis (**Figure 5A**) showed that after *S. japonicum* infection, as expected, Ikzf2 was expressed in the nucleus of ICOS^+^ Th cells, but not in the nucleus of ICOS^−^ Th cells. Ikzf2 was not expressed in the cytoplasm of both ICOS^+^ Th and ICOS^−^ Th cells. It indicated that Ikzf2 entered into the ICOS^+^ Th nucleus after *S. japonicum* infection. Then, we detected whether Ikzf2 entered the ICOS^+^ Th nucleus and directly bound to the promoter of ICOS to play a regulatory role after infection. In order to obtain enough target cells for the ChIP experiment, the splenocytes were stimulated with anti-CD3 and anti-CD28 antibodies, and ICOS^+^ and ICOS^−^ Th cells were selected by magnetic bead sorting. The purity of the sorted cells is shown in **Figure 5B**. In order to obtain 150–900 bp DNA fragments for subsequent ChIP experiments, a chromatin shearing kit was used to process the target cells. The results of chromatin shearing efficiency analysis are shown in **Figure 5C**. qRT-PCR was used to detect the efficiency of immunoprecipitation with different antibodies. The results (**Figure 5D**) showed that in the samples treated with normal IgG, the efficiency of immunoprecipitation with the ICOS promoter was low and there was no statistical difference between the ICOS^+^ group and the ICOS^−^ group (*P* > 0.05). Simultaneously, histone H3 antibodies were used for immunoprecipitation to ensure the accuracy of the experiment. In the Ikzf2 antibody immunoprecipitation samples, the efficiency of immunoprecipitation with the ICOS promoter in the ICOS^+^ group was significantly higher than that in the ICOS^−^ group (*P* < 0.01).

RETRACTED

**Figure 5:** Ikzf2 transferred into the nucleus of ICOS^+^ Th cells and bound to the promoter *icos* gene after *S. japonicum* infection. **(A)** Five to 6 weeks after *S. japonicum* infection, splenocytes were isolated and stained by different fluorescence-labeled antibodies. CD4^+^ ICOS^+^ T cells and CD4^+^ ICOS^−^ T cells were sorted by FACS, respectively. After the separation of nucleoplasmic proteins, the distribution of Ikzf2 was detected by Western blotting. Tubulin and histone H3 were used as cytoplasm and nucleus controls. **(B)** CD4^+^ T cells were stimulated with CD3 and CD28 mAb for 24 h, and ICOS^+^ **^/^** ^−^ Th cells were selected by magnetic bead sorting. The expression of ICOS was detected by flow cytometry. **(C)** The DNA fragments of the sorted cells treated with the chromatin shearing kit were analyzed by DNA electrophoresis. The sheared length of DNA should be about 150–900 bp. **(D)** ChIP results were obtained by qRT-PCR. Anti-Ikzf2 mAb, positive control histone H3 rabbit mAb, and negative control normal rabbit IgG were added to pull down the promoter of ICOS, respectively. Percent Input = 2% × 2^(C[T] 2%Input Sample − C[T] IP Sample)^. Data were shown as three samples in each group from one representative experiment, and experiments were repeated three times with similar results. **(E)** HEK293T cells were transfected with ICOS promoter reporter plasmids containing the firefly luciferase and the *renilla luciferase* gene. Simultaneously, 500 ng of Ikzf2-flag plasmids and empty vectors were transfected into HEK293T cells. Twenty-four hours after transfection, IKZF2 expression were detected by Western blot. β-Actin was used as an internal reference protein. **(F)** The remaining cell lysates were used for the DLR test. The ratio of firefly luciferase activity to Renilla luciferase activity was converted to relative luciferase activity. The means are from three independent experiments and the error bars are SD. **P < 0.01, and *ns*, not significant (*P* > 0.05).

RETRACTED

To further support this hypothesis, PmirGLO plasmid containing the *ICOS promoter*, *luciferase*, and *hRluc* genes; pCDNA3.1(+) plasmid expressing the *Ikzf2* gene; and the corresponding empty vector were constructed. These plasmids were transfected into 293T cells. Firstly, the protein expressions of the plasmids were verified by Western blot. Twenty-four hours after transfection, pCDNA3.1(+) plasmid expressing the *Ikzf2* gene was successfully transfected into 293T cells and expressed (**Figure 5E**). Then, dual-luciferase reporter assays were performed. Compared with the group-transfected empty vector, the group-transfected Ikzf2 plasmid resulted in a strong induction of ICOS promoter activity (*P* < 0.01, **Figure 5F**). These data showed that Ikzf2 could bind to the ICOS promoter and regulate ICOS expression.

In summary, from the results of our study, it was demonstrated that Ikzf2 was transferred into the nucleus of Th cells after *S. japonicum* infection and could bind to the promoter of ICOS to launch the expression of ICOS.

## Discussion

*S. japonicum* infection could induce serious systemic inflammation in mice (**Supplementary Figure 1**). Recent researches have demonstrated that ICOS, as a co-stimulatory molecule, can not only regulate the functions of Th cells and effector T cells but also induce B-cell differentiation and antibody production (18). In this study, as shown in **Figure 1**, after *S. japonicum* infection, the number of lymphocytes in the spleen increased significantly (*P* < 0.01). The ICOS molecule in the splenocytes from *S. japonicum*-infected mice increased significantly in both mRNA and protein levels (*P* < 0.05). It implied that ICOS might play a pivotal role in the course of *S. japonicum* infection-induced diseases. Similar results were also reported in rheumatoid arthritis patients (19). Multiple studies have indicated that ICOS is expressed not only on CD4^+^ Th cells but also on CD8^+^ T cells (20) and CD19^+^ B cells (21). The results of this study indicated that the percentage of ICOS^+^ cells increased significantly on CD4^+^ Th cells and CD19^+^ B cells after *S. japonicum* infection (*P* < 0.05), whereas there was no significant difference in the ICOS changes of CD8^+^ T cells. Similar results were found in the liver and lungs of *S. japonicum*-infected mice (**Supplementary Figure 2**). Studies have shown that there is no significant difference in liver granuloma and fibrosis caused by S*chistosoma* between wild-type and CD8^+^ T-cell knockout mice. These results suggested that CD8^+^ T cells are not the key players in regulating the immune response during *S. japonicum* infection. The further experiment indicated that the increase of ICOS expression mainly distributed in splenic CD4^+^ Th cells, which increased rapidly 1 week after infection, reached a peak at weeks 4–6. It implied that ICOS mediates *S. japonicum* infection-induced immune response mainly through mediating the function of CD4^+^ Th cells (22).

RETRACTED

ICOS appears to costimulate distinct effector functions in different immune responses. For example, ICOS molecules can promote the activation and function of Th cells during anti-OX40-driven tumor immune responses (23). Treatment with ICOS antibody can weaken symptoms and prolong survival in the chronic graft-*versus*-host disease (GVHD) model (24). Herein, comparison of ICOS^+^ Th cells and ICOS^−^ Th cells showed that more ICOS^+^ Th cells expressed CD69, and less of them expressed CD62L. Since CD69 and CD62L were classic markers reflecting T-cell activation (25, 26), it was demonstrated that ICOS could help Th cell activation in the course of *S. japonicum* infection. Previous studies reported that Th cells promoted B-cell differentiation and germinal center formation and plasma cell differentiation through CD40L (12) and CXCR5 (27). We demonstrated that both CD40L and CXCR5 were significantly increased in ICOS^+^ Th cells after *S. japonicum* infection, which suggested that ICOS^+^ Th cells possessed strong abilities in promoting B-cell-mediated immune response in *S. japonicum*-infected mice. RNA sequencing results also showed that the expression of activating molecules (CD69, CXCR5, and CD40L) increased in the ICOS^+^ cells (**Figure 3**).

Cytokine release is an important manner for Th cells to mediate the immune response. IL-4 is a cytokine secreted by activated T cells and promotes the differentiation and maturation of B cells (28–30). IFN-γ is a key factor that drives cellular immunity and can coordinate the functions of immune cells to enhance the immune response to pathogen infection and cancer (31, 32). Studies indicated that Th cells could mediate the *Schistosoma* infection-induced immune response by secreting IL-4, IL-5, IL-9, and so on (33). The intracellular cytokine staining results showed that more cytokines could be released by ICOS^+^ Th cells. Although Th cells in mice infected with *S. japonicum* were dominated by Th2 immunity (34), we found that more ICOS^+^ Th cells can express IL-4 and IFN-γ. These results were verified by RNA sequencing (**Figure 3**). Then, GO and KEGG analyses suggested that ICOS was involved in the differentiation and maturation of immune cells, cytokine production, and other signaling pathways. All these results suggested that ICOS played a crucial role in maintaining both Th1 and Th2 immunity (35).

RETRACTED

ICOS is a key player in the inflammatory diseases, but the molecular regulation mechanism is not well known. According to reported studies, the enhanced glycolytic activity due to Von Hippel-Lindau gene deficiency was involved in the epigenetic regulation of ICOS expression, and glycolytic enzyme GAPDH was the key target for the reduced ICOS expression *via* m^6^A modification by using an RNA interference screen (36). Choi J and his colleagues reported that expression of ICOS and CD200 in CXCR5^+^ Th cells was upregulated in the absence of Runx2 and Runx3 (37). Similarly, ICOS expression is modestly increased in Bcl-6-lentiviral vector (LV)-treated CD4^+^ T cells from human tonsil. ICOS expression was higher in Bcl-6-LV and maf-LV co-treated Th cells (38). The expression of Nfatc1 was significantly increased and accompanied by an increase in ICOS expression in patients with nonsmall cell lung cancer (39). RGS16 act as oncogenes and promote malignancy progression of many human cancers (40). It was reported that RGS16 could restrict the proinflammatory response of monocytes (41). Our study showed that RGS16 was the top ranked transcription factor which increased the expression in ICOS^+^ Th cell (**Figure 4A**). It suggested that RGS16 might play an important role in regulating ICOS expression.

Ikaros zinc finger (Ikzf) transcription factors were recently reported to be important transcription factors that regulated lymphocyte development and differentiation (42), and were significantly increased in ICOS^+^ cells (43). Ikzf2 (Helios), a member of the Ikaros transcription regulator family, is associated with Th cell differentiation (44, 45). Results (**Figures 4A–D**) showed that the expression of Ikzf2 increased significantly in ICOS^+^ Th cells at both the mRNA and protein levels (*P* < 0.05). It suggested that *Ikzf2* might be the main gene to regulate the expression of ICOS in Th cells from *S. japonicum-*infected mice. Furthermore, Western blot results demonstrated that Ikzf2 entered into the nucleus of ICOS^+^ Th cells, but not in the ICOS^−^ nucleus (**Figure 5A**). It suggested that Ikzf2 could bind to the promoter of ICOS.

ChIP exploits the specific interactions between DNA and DNA-associated proteins. It can be used to examine a wide range of experimental parameters (46). A number of proteins bound at the same genomic location can identify a multiprotein chromatin complex where several proteins work together to regulate gene transcription or chromatin configuration (47–49). In this study, ChIP was done, and qRT-PCR was used to detect the efficiency of immunoprecipitation. Results showed that Ikzf2 could bind to the promoter of ICOS directly in the nucleus of ICOS^+^ Th cells (**Figures 5B–D**). Dual-luciferase reporter assays are an important means to explore the specific sequence binding of transcription factors and their target promoters (50, 51). Moreover, our data (**Figures 5E, F**) show that Ikzf2 resulted in strong induction of ICOS promoter activity, too. All these results illustrated that Ikzf2 was the key transcription factor that is responsible for the expression of ICOS on CD4^+^ T cells in the course of *S. japonicum*-induced splenomegalia.

RETRACTED

In conclusion, our study found that transcription factor Ikzf2 was the key regulating molecule, which could bind to the promoter of ICOS in Th cells directly to launch the expression of ICOS, and ICOS expressing CD4^+^ Th cells played an important role in regulating host immunity after *S. japonicum* infection.

## Data Availability Statement

The datasets presented in this study can be found in online repositories. Transcriptome-seq raw sequences deposited in Sequence Read Archive (SRA) are available at NCBI SRA portal with SRA IDs: SRR14038879 and SRR14038945.

## Ethics Statement

The animal study was reviewed and approved by the Institutional Animal Care and Use Committee of Guangzhou Medical University (S2020-055).

## Author Contributions

SX, HW, and AP performed most of the experiments and analyzed the data with support from JH. AX, JL, CF, and FS performed the animal experiments. HH and HX performed the parasite infection experiment. QY contributed to scientific planning. XP and JH designed the study. XT and JH wrote the manuscript. All authors contributed to the article and approved the submitted version.

## Funding

This research was supported by grants from the Natural Science Foundation of China (81771696, 81802024), the Natural Science Foundation of Guangdong Province (2020A1515010251, 2021A1515011032, 2018A030313217), and Guangzhou Science and Technology Project (202002030082).

## Conflict of Interest

The authors declare that the research was conducted in the absence of any commercial or financial relationships that could be construed as a potential conflict of interest.

## Publisher’s Note

All claims expressed in this article are solely those of the authors and do not necessarily represent those of their affiliated organizations, or those of the publisher, the editors and the reviewers. Any product that may be evaluated in this article, or claim that may be made by its manufacturer, is not guaranteed or endorsed by the publisher.
